The article "Prevalence and Morphology of C-Shaped Canals in Mandibular First and Second Molars of an Iranian Population: A Cone-Beam Computed Tomography Assessment" was published in 2023. Journal: Scanning.

# Prevalence and Morphology of C-Shaped Canals in Mandibular First and Second Molars of an Iranian Population: A Cone-Beam Computed Tomography Assessment

**DOI:** 10.1155/2023/5628707

**Published:** 2023-10-03

**Authors:** Ahmad Nouroloyouni, Neda Moradi, Amin Salem Milani, Sara Noorolouny, Nazila Ghoreishi Amin

**Affiliations:** ^1^Department of Endodontics, School of Dentistry, Ardabil University of Medical Science, Ardabil, Iran; ^2^Department of Endodontics, School of Dentistry, Tabriz University of Medical Science, Tabriz, Iran; ^3^Department of Pediatric Dentistry, Ardabil University of Medical Science, Ardabil, Iran; ^4^Department of Radiology, University of Southern California, Los Angeles, USA

## Abstract

**Objectives:**

The complex anatomy of C-shaped canals poses challenges for clinicians compared to teeth with normal root canal anatomy. This study is aimed at evaluating the frequency and morphology of C-shaped canals in the mandibular first and second molars among an Iranian population using cone-beam computed tomography (CBCT).

**Materials and Methods:**

This cross-sectional study evaluated 369 CBCT scans from the archives of a radiology clinic in Ardabil, Iran. The sample included 248 mandibular first molars and 478 mandibular second molars. The presence of C-shaped canals and their classification, according to Fan et al., were evaluated at four levels: orifice, coronal, middle, and apical. Prevalence based on gender and tooth type was also assessed.

**Results:**

A total of 199 (53.9%) males and 170 (46.1%) females were evaluated. C-shaped canals were found in 11 (8 males/3 females) out of 248 (4.4%) first molars and in 20 (11 males/9 females) out of 478 (3.7%) second molars. The C2 configuration was most prevalent in the orifice, coronal, and middle levels of both molar types, while C3 and C4 morphologies were most commonly found apically in the second and first molars, respectively. A significant difference in configuration was found only at the coronal level between molar types. A significant association between gender and configuration was observed only at the orifice level of the second molars. No other significant differences were found (*P* > 0.05).

**Conclusion:**

C-shaped canal configurations should be expected in 4.4% of mandibular first molars and 3.7% of the second molars in this Iranian population, with a predominance of the C2 configuration in the orifice, coronal, and middle levels.

## 1. Introduction

Comprehensive knowledge of root canal anatomy is essential for successfully cleaning and filling the root canal system [1]. Also, it is important for clinicians to have adequate knowledge about anatomical variations and root canal abnormalities because it has been proven that the presence of a single conical canal with one apical foramen is an exception rather than the rule [2].

Root formation commences with the apical proliferation of epithelial cells from Hertwig's epithelial root sheath [3], which acts as a template for root development. The pattern of cell proliferation in the sheath is genetically determined, and it determines the width or narrowness, straightness or curvature, and length or shortness of the root [4].

Mandibular first and second molars can exhibit variations in root canal anatomy. C-shaped canals are prevalent in them, with fins and webs connecting the canals [5]. Such irregular areas contain residual soft tissue, which is often inflamed and infected. These areas are difficult to access, and their debridement is complex. Thus, they can cause problems during root canal treatments [6].

C-shaped canals were first reported in 1979 [7]. The majority of C-shaped canals occur in mandibular second molars. However, they have also been reported in the mandibular first molars, maxillary first and second molars, and mandibular premolars [8]. The prevalence of C-shaped canals varies among different races and populations [9]. C-shaped canals have a high prevalence in Asian countries [10]. A C-shaped canal forms due to the fusion of the mesial and distal roots on the buccal or lingual root surface. This fusion is often incomplete, and the two root canals are connected by a fin [11].

Due to the complex anatomy of C-shaped canals, teeth with C-shaped canals undoubtedly pose more of a challenge to clinicians than those with normal root canal anatomy [6]. Therefore, having comprehensive knowledge about the type and prevalence of this anatomical variation may help reduce the risk of endodontic treatment failure in these teeth.

Melton et al. [12] demonstrated that the shape of the canal in C-shaped canals may vary along the length of the root. They also found that the clinical appearance of the crown or orifice shape is not a highly reliable indicator of the canal shape. They proposed a classification system for C-shaped canals. Also, Fan et al. [13] evaluated the correlation between radiographic manifestations of C-shaped mandibular second molars and the cross-sectional shape of the root canal system. Accordingly, the radiographic manifestations were categorized.

Cone-beam computed tomography (CBCT) and microcomputed tomography (CT) enable noninvasive in vivo assessments of the effects of race, age, and gender on anatomy [14]. They also enable detailed qualitative and quantitative evaluation of specific anatomical characteristics [14]. CBCT accurately depicts pulp chamber/canal morphology in three dimensions, often surpassing the capabilities of intraoral radiography. It allows evaluation of the canal path in axial, coronal, and sagittal planes for treatment planning [15]. Compared to CT, CBCT offers higher accuracy and resolution, faster scan times, and lower patient radiation doses, making it a valuable tool for dental applications [16]. CBCT has been used in complicated cases [17] and provides an excellent educational tool with numerous benefits. Analysis of existing CBCT scans can identify weaknesses in clinical practice, facilitating targeted learning interventions [18, 19].

A recent study examined endodontic errors and mandibular molar anatomy in this population, but it lacked information on C-shaped canals [19]. Considering the significance of comprehensively understanding the prevalence and morphology of C-shaped canals, our objective was to fill this research gap by assessing the prevalence and morphology of C-shaped canals in mandibular molars within the Iranian population. Our findings provide clinically useful data on the frequency and morphology of this anatomical variation, which can be used to inform endodontic treatment planning and technique.

## 2. Materials and Methods

### 2.1. Ethical Consideration

The study was approved by the ethics committee of Ardabil University of Medical Sciences (IR.ARUMS.REC.1398.366). Patients consented to the use of their CBCT scans for research purposes at the time of imaging.

### 2.2. Data Collection Procedure

This cross-sectional study was conducted on CBCT scans retrieved from the archive of a radiology clinic in Ardabil City, Iran, using convenience sampling. The CBCT scans were obtained between 2017 and 2019 for diagnostic purposes or preoperative assessments, unrelated to this study. The sample size was calculated to be 369 using Cochrane's formula for sample size calculation.

The inclusion criteria were high-quality CBCT scans that visualized at least one mandibular molar with fully developed roots, without any periapical lesion, deep carious lesion, previous endodontic treatment, or presence of intracanal posts, deep fillings, and crowns. All CBCT scans were obtained using the NewTom GiANO (Verona, Italy) CBCT scanner with settings of 90 kVp, 3 mA, voxel size of 0.2 mm, a field of view of 11 cm by 13 cm, and an exposure time of 9 seconds. The scans were performed by an oral and maxillofacial radiologist. NNT software (NewTom 5G, QR, Verona, Italy) was used to evaluate the images. If necessary, the image contrast and brightness were adjusted to achieve optimal visualization.

The present study is aimed at determining the prevalence and morphology of C-shaped root canals in mandibular first and second molars. Prevalence based on gender and tooth type was also evaluated. A C-shaped canal was diagnosed if it had all the three characteristics defined by Fan et al. [13] as follows:

(ii) Fusion of roots along their entire length
(iii) Presence of a longitudinal groove in the buccal or lingual surface
(iiii) At least one section of the canal must show a C-shaped canal

For each eligible tooth, the C-shaped canal structure was categorized into the following classes according to Fan et al. (Figure 1) [13]. Canals were evaluated at distinct four cross-sectional levels: O (orifice); C (coronal), 2 mm from the root canal orifice; M (middle), at the middle of the root canal length; and A (apical), 2 mm from the apical foramen [20].

C1: Continuous C-shaped

C2: Canal shape is in the form of a semicolon, due to discontinuation of the “C” outline. However, the *α* or *β* should not be <60 degrees. The *α* or *β* angles could be determined according to Figure 2. [5]

C3: Presence of 2 or 3 separate canals, and both *α* and *β* are <60 degrees

C4: Presence of one round or oval canal

C5: Absence of canal lumen [5]

A senior dental student, who was trained and calibrated, evaluated the CBCT scans under the supervision of an endodontist and an oral and maxillofacial radiologist. The teeth on CBCT images were evaluated in the sagittal, coronal, and axial planes using NNT software (NewTom 5G, QR, Verona, Italy). To ensure the validity and reliability of the assessments, 25% of the CBCT scans were randomly selected and reevaluated by the supervising oral and maxillofacial radiologist, as well as an endodontist. Additionally, in order to evaluate intraexaminer reliability, 25% of the CBCT scans were assessed by the senior dental student 10 days after their initial evaluation. The agreement between the findings in the first and second observations was assessed using Cohen's kappa, which resulted in a fully reliable agreement (kappa = 0.96).

### 2.3. Statistical Analysis

SPSS version 25 (SPSS Inc., Chicago, IL, USA) was used to analyze the data. The frequency and proportion of C-shaped canals were compared in mandibular first and second molars and in different genders using the Monte Carlo tests at 0.05 level of significance.

## 3. Results

### 3.1. Mandibular First Molars

Out of 369 patients, 187 did not have mandibular first molars. Out of 182 with mandibular first molars, 116 had one molar and 66 had both mandibular first molars. Of the 248 mandibular first molars, 11 teeth (4.4%) had a C-shaped canal.

### 3.2. Mandibular Second Molars

Out of 369 patients, 39 did not have mandibular second molars. Of the 330 patients with mandibular second molars, 182 had one, and 148 had both mandibular second molars. Of the mandibular second molars, 20 teeth (3.7%) had C-shaped canals.

### 3.3. Correlation of Tooth Type (Mandibular First/Second Molar) with C-Shaped Canal Types at Different Levels

Table 1 represents the frequency of different types of C-shaped canals of mandibular first and second molars at various levels.

The C2 configuration was most prevalent in the orifice, coronal, and middle levels of both molar types, while C3 and C4 morphologies were most commonly found apically in the second and first molars, respectively. The Monte Carlo test revealed a statistically significant correlation between the occurrence of various types of C-shaped canals and the tooth type (mandibular first/second molar), only at the coronal level (*P* = 0.011), as shown in Table 1.

### 3.4. Correlation of Gender with C-Shaped Canals in Different Levels of Mandibular First and Second Molars

Of the 369 patients, 199 (53.9%) were males and 170 (46.1%) were females. Of the 11 C-shaped mandibular first molars, 8 were males and 3 were females. Additionally, out of the 20 C-shaped mandibular second molars, 11 were males and 9 were females.

The frequency of different types of C-shaped canals in different genders at various levels in each tooth type is presented in Tables 2 and 3.

There is no statistically significant connection between the type of C-shaped canal and gender for either of the two types of teeth studied at the four root levels, except for the second molar at the orifice level (*P* value > 0.05).

### 3.5. Correlation of Different Types of C-Shaped Canals of Different Genders and Different Tooth Types in Different Levels

The findings from Table 3, based on the Monte Carlo test, indicate that there is no statistically significant relationship between the prevalence of C-shaped canal types in the two types of teeth being studied and the patient's gender at any of the four root levels investigated (*P* value > 0.05).

## 4. Discussion

The complex anatomy of C-shaped canals, including the difficult-to-clean fin areas, poses challenges for clinicians compared to teeth with normal canal anatomy [6]. Comprehensive knowledge regarding the prevalence and variations of this anatomy can help reduce the occurrence of endodontic treatment failures in these teeth. Recent research has examined endodontic errors and anatomical characteristics of mandibular molars in an Iranian population [19]. However, information on C-shaped canals in this population is lacking. Our study is aimed at addressing this gap by evaluating the prevalence and morphology of C-shaped anatomy in mandibular molars within a specific Iranian population. This study provides clinically useful data on the frequency of this anatomical variation, which can help improve endodontic treatment planning and technique in this patient population.

The present study provides detailed information on the C-shaped morphology in mandibular first and second molars using CBCT in an Iranian population. Several techniques exist for assessing root canal anatomy, including tooth clearing, resin impressions, and radiography. However, two-dimensional radiographs may not clearly visualize C-shaped canals because of root overlap. Micro-CT has also been utilized, but it is not clinically applicable [21]. CBCT was used in this study because it does not require sectioning or damaging teeth and can be applied clinically [21]. We analyzed existing CBCT scans taken for other diagnostic or treatment purposes, which provided an excellent noninvasive means of obtaining anatomical information [17, 19].

The root morphology of the Iranian population differed from that of other populations in our study. The present results showed that 4.4% of mandibular first molars had a C-shaped canal configuration. However, most previous studies have reported lower rates in the first molars compared to our findings. Celikten et al. [22] found that only 2 out of 384 first molars in the Turkish population had C-shaped canals. Another study conducted on a Portuguese population (695 teeth) reported that 0.6% of the first molars had C-shaped canals, as classified by the Fan classification [23]. A study using CBCT on 1020 Israeli patients revealed that 0.16% of 1465 first molars and 4.6% of 1229 second molars had C-shaped canals [24]. The majority of studies report a very low prevalence of C-shaped canals in the first molars. The higher frequency observed in our study may be attributed to genetic variations among the populations that were examined. The only study that reported a higher rate of C-shaped configurations in mandibular first molars was conducted by Vaz de Azevedo et al. [25]. They found frequencies of 24.01% and 21.32% for C-shaped configurations in the first and second mandibular molars, respectively.

The present results showed that 3.7% of the second molars had a C-shaped canal configuration. Previous studies have reported varying prevalence rates of C-shaped canals in mandibular molars. Some studies, especially in Eastern Asia, have reported high frequency rates for C-shaped canals. Jin et al. [26] demonstrated that 44.5% of the teeth in their study population had a C-shaped canal. The reported value in their study is more than 10 times higher than the rate in the present study. This controversy may be attributed to racial differences among the study populations.  Table 4 provides a comprehensive overview of the results from diverse studies conducted in various geographical regions.

Melton et al. [12] showed that the shape of the canal may vary along the length of the root in C-shaped canals, and the clinical form of the crown or orifice shape is not highly reliable for predicting the shape of the canal. Frequencies of different configurations at cross-sectional levels have also been shown to vary among populations. In our study, canals were evaluated at four distinct cross-sectional levels: orifice, coronal, middle, and apical. In our study, the configuration of C2 had the highest prevalence in both the mandibular first and second molars at the orifice, coronal, and middle levels. In the apical level, C3 and C4 configurations were more prevalent in mandibular second and first molars, respectively. Several previous studies by Kim et al. [20], Fan et al. [5], Zheng et al. [33], and Seo et al. [34] have reported that the C1 type was most prevalent coronally at the orifice level (66%), while the C3 type predominated apically (56%). Additionally, Kim et al. [20] observed that the frequency of C1 and C2 morphologies decreased from the orifice to the apex, while C3 and C4 became more common apically. The present results confirm the general trends described in earlier studies, showing a transition from C2 coronally to more C3 and C4 apically in both the mandibular first and second molars with C-shaped canals.

Kim et al. [20] previously stated that gender should be considered when determining root canal morphology before treatment. However, the present study found no statistically significant association between the C-shaped canal type and gender at the examined root levels in both types of mandibular molars (Table 3). The only exception was at the level of the orifice of the second molars, where the canal configuration differed by gender (Table 2). These findings align with several other studies by Zheng et al. [33], Helvacioglu-Yigit and Sinanoglu [35], and Ladeira et al. [21] that also reported nonsignificant relationships between the occurrence of C-shaped canals and gender. In contrast, Kim et al. [20] found a significantly higher prevalence in females (47%) compared to males (32%). A study in Venezuela documented slightly higher rates among males, although the difference was not statistically significant [31]. These contradictory results may arise from differences in sample sizes and the ethnic backgrounds of participants across studies. Further large-scale research is needed to clarify potential gender differences in the prevalence and morphology of C-shaped canals.

### 4.1. Clinical Relevance

C-shaped canals are considered to be one of the greatest anatomical challenges in endodontics, making the clinical significance of these findings undeniable. The complex morphology of these canals, characterized by narrow and irregular areas, can serve as a reservoir for soft tissues, microorganisms, and dentinal detritus. These areas may not be completely removed during treatment, which can diminish its efficacy. The difficulty of detecting C-shaped canals by clinicians is greater than anticipated. Although the presence of fused molar roots may indicate the presence of C-shaped canals, it is important to note that the radiographic appearance of two distinct roots does not necessarily rule out the possibility of C-shaped canals [36].

According to the high prevalence of C-shaped canals, especially in mandibular first molars, in the population of this study, it is recommended that when a clinician suspects the presence of C-shaped canals, they should use CBCT images and an operating microscope. CBCT images act as a map, and the magnification provided by the microscope helps in detecting additional canals [37, 38].

### 4.2. Limitations of the Study and Suggestions for Future Studies

One limitation of the current study was the lack of access to the age of the patients. Research has shown that due to secondary dentin deposition in the root canal, the root canal space can be eventually obliterated, obstructing the radiographic appearance of these anatomically complex structures. The incidence of C-shaped canal morphology decreases with age [30, 39]. As another case study with sufficient data availability, it is suggested to include the impact of age in the final outcome.

Due to the rare occurrence of C-shaped canals in mandibular first molars, limited research has been conducted on this topic. In light of the results of the present study and the likelihood of a higher prevalence of C-shaped morphology in mandibular first molars in certain regions, such as our study population, it is suggested that further research be conducted in this area.

## 5. Conclusion

C-shaped canal configurations were found in 4.4% of mandibular first molars and 3.7% of the second molars in this Iranian population. The C2 configuration was predominantly observed in the orifice, coronal, and middle levels, while C3 and C4 morphologies were most common apically in the second and first molars, respectively. The present study found no statistically significant association between the C-shaped canal type and gender at most of the examined root levels in both types of mandibular molars. The only exception was at the level of the orifice of the second molars, where the canal configuration differed by gender.

## Figures and Tables

**Figure 1:** C-shaped canal structure categories [13].

**Figure 2:** Measurements of the angles *α* and *β* to differentiate the C2 and C3 canal configurations: A and B: ends of one canal cross-section; C and D: ends of the other canal cross-section; M: middle point of line AD; *α*: angle between line AM and line BM; *β*: angle between line CM and line DM. (a) C2 canal configuration, angle *β* > 60°. (b) C3 canal configuration, *α* < 60°, *β* < 60° [5].

**Table 1:** Frequency of different types of C-shaped canals of mandibular first and second molars in different levels.

Type of C-shaped canal	Orifice		Coronal		Middle		Apical	
	First molar	Second molar	First molar	Second molar	First molar	Second molar	First molar	Second molar
C1	2 (6.5%)	6 (19.4%)	0	3 (9.7%)	0	1 (3.2%)	0	1 (3.2%)
C2	9 (29.0%)	8 (25.8%)	11 (35.5%)	9 (29.0%)	7 (22.6%)	9 (29.0%)	4 (12.9%)	4 (12.9%)
C3	0	4 (12.9%)	0	6 (19.4%)	4 (12.9%)	7 (22.6%)	2 (6.5%)	8 (25.8%)
C4	0	2 (6.5%)	0	2 (6.5%)	0	3 (9.7%)	5 (16.1%)	7 (22.6%)
*P* value^∗^	0.085		0.011		0.568		0.505	

^∗^ *P* < 0.05 was considered statistically significant.

**Table 2:** The frequency of different types of C-shaped canals in different levels and in different genders in mandibular first and second molars.

Tooth type	Type of C-shaped canal	Orifice		Coronal		Middle		Apical	
		Male	Female	Male	Female	Male	Female	Male	Female
First molar	C1	2 (18.2%)	0	0	0	0	0	0	0
	C2	6 (54.5%)	3 (27.3%)	8 (72.7%)	3 (27.3%)	5 (45.5%)	2 (18.2%)	4 (36.4%)	0
	C3	0	0	0	0	3 (27.3%)	1 (9.1%)	1 (9.1%)	1 (9.1%)
	C4	0	0	0	0	0	0	3 (27.3%)	2 (18.2%)
	*P* value^∗^	0.566		—		1.000		0.333	

Second molar	C1	1 (5.0%)	5 (25.0%)	0	3 (15.0%)	0	1 (5.0%)	0	1 (5.0%)
	C2	4 (20.0%)	4 (20.0%)	4 (20.0%)	5 (25.0%)	4 (20.0%)	5 (25.0%)	2 (10%)	2 (10%)
	C3	4 (20.0%)	0	5 (25.0%)	1 (5.0%)	5 (25.0%)	2 (10%)	4 (20.0%)	4 (20.0%)
	C4	2 (10.0%)	0	2 (10%)	0	2 (10%)	1 (5.0%)	5 (25.0%)	2 (10%)
	*P* value	0.022		0.055		0.525		0.650	

^∗^ *P* < 0.05 was considered statistically significant.

**Table 3:** Frequency of different types of C-shaped canals of different genders and different tooth types in different levels.

Root level	Tooth type	C1		C2		C3		C4	
		Male	Female	Male	Female	Male	Female	Male	Female
Orifice	6	2 (25%)	0	6 (35.3%)	3 (17.6%)	0	0	0	0
	7	1 (12.5%)	5 (62.5%)	4 (23.5%)	4 (23.5%)	4 (100%)	0	2 (100%)	0
	*P* value^∗^	0.109		0.629		—		—	

Coronal	6	0	0	8 (40%)	3 (15%)	0	0	0	0
	7	0	3 (100%)	4 (20%)	5 (25%)	5 (83.3%)	1 (16.7%)	2 (100%)	0
	*P* value	—		.357		—		—	

Middle	6	0	0	5 (31.2%)	2 (12.5%)	3 (27.3%)	1 (9.1%)	0	0
	7	0	1 (100%)	4 (25%)	5 (31.2%)	5 (45.5%)	2 (18.2%)	2 (66.7%)	1 (33.3%)
	*P* value	—		.350		1.000		—	

Apical	6	0	0	4 (50%)	0	1 (10%)	1 (10%)	3 (25%)	2 (16.7%)
	7	0	1 (100%)	2 (25%)	2 (25%)	4 (40%)	4 (40%)	5 (41.7%)	2 (16.7%)
	*P* value	—		0.428		1.000		1.000	

^∗^ *P* < 0.05 was considered statistically significant.

**Table 4:** Prevalence of C-shaped canal configurations observed in mandibular molars, as reported in the previous studies.

Author (year)	Region	Tooth type	Number of teeth	Prevalence of C-shaped configuration
Madani et al. [27]	Iran	Man.^∗^ 1st molar	147	1.2%
		Man. 2nd molar	154	17.6%

Alfawaz et al. [28]	Saudi Arabia	Man. 1st molar	529	0.19%
		Man. 2nd molar	681	9.1%

Martins et al. [23]	Portugal	Man. 1st molar	695	0.6%
		Man. 2nd molar	1088	8.5%

Shemesh et al. [24]	Israel	Man. 1st molar	1229	0.16%
		Man. 2nd molar	1465	4.6%

Vaz de Azevedo et al. [25]	Brazil	Man. 1st molar	389	23%
		Man. 2nd molar	422	21.32%

Demirbuga et al. [29]	Turkey	Man. 1st molar	823	0.85%
		Man. 2nd molar	925	4.1%

Celikten et al. [22]	Turkey Cypriot	Man. 1st molar	384	0.5%
		Man. 2nd molar	421	1.9%

von Zuben et al. [9]	United States	Man. 2nd molar	400	11.3%
	South Africa		400	9.3%
	Mexico		400	14.2%

Abdalrahman et al. [30]	Iraq	Man. 2nd molar	368	17.4%

Gomez et al. [31]	Venezuela	Man. 2nd molar	190	19.5%

Park et al. [32]	Korea	Man. 2nd molar	710	41.3

Present study	Iran	Man. 1st molar	248	4.4%
		Man. 2nd molar	478	3.7%

^∗^Mandibular.

## Data Availability

The data used to support the findings of this study were supplied by the corresponding author under license, and data will be available on request up to one year after publication. Requests for access to these data should be made to the corresponding author.
